# Mathematical Analysis of Application of a Three-Dimensional Printing Fixator in the Fracture of Multiple Ribs

**DOI:** 10.1155/2021/5626228

**Published:** 2021-10-01

**Authors:** Zhigong Zhang, Jinsong Yang, Haoyu Zou, Wen Wang, Xiangyi Wu, Xiaojuan Lin

**Affiliations:** ^1^Department of Cardiothoracic Surgery, Hunan Provincial People's Hospital (The First-Affiliated Hospital of Hunan Normal University), Changsha 410005, China; ^2^Department of Paediatrics, Hunan Provincial People's Hospital (The First-Affiliated Hospital of Hunan Normal University), Changsha 410005, China

## Abstract

Data were obtained from 66 clinical patients. The patients were divided into a non-3D printing group (control group) and a 3D printing group (intervention group) in a 1 : 1 ratio, with 33 patients in each group. The information including gender, age, incision length, number of surgical roots, bleeding volume, operation time, and intraoperative blood transfusion was collected for SPSS analysis. The results showed the following: (1) The paired *t*-test was used to test the difference of experimental data. There was a significant difference of 0.01 between the incision length/surgical root number in the intervention group and the incision length/surgical root number in the control group. The incision length/surgical root number in the intervention group was significantly lower than that in the control group. (2) Surgical time, intraoperative blood transfusion, age, and incision length/surgical root number in the intervention group had a significant positive impact on the amount of bleeding. Gender did not affect the amount of bleeding. (3) A total of 1 item of operation time in the intervention group had a significant positive impact on intraoperative blood transfusion. (4) The incision length/number of surgical roots in the intervention group had a noteworthy negative impact on blood transfusion during the operation.

## 1. Introduction

Three-dimensional printing technology has been widely used in medicine [1–3]. At present, the 3D auxiliary fixator preshapes length, angle, and other three-dimensional shapes of the fracture fixator for patients preoperatively according to the conditions of bones, nerves, and blood vessels of patients. Based on a large amount of reported evidence, the application of three-dimensional printing technology in fracture surgery can effectively reduce the incision length [4], shorten the operation time [5], reduce complications such as hemorrhage and nerve injury [6], and postoperative intercostal neuralgia [7, 8] and finally reduce the mortality rate of trauma patients.

There are a large number of studies using mathematical methods for relevant statistical analysis [9–11]. Avşar and Ün [12] have studied a 3D visualization tool, which can automatically generate the real model of a 3D fixator according to the human condition. Herath and Epaarachchi [13] used the CAD software to design the geometric model for the transverse fracture and fracture of the male tibia and finally printed in 3D. Abdul Wahab et al. [14] studied the double cross-locking structure of the 3D fixator at the fracture site and the external fixator and considered it to be optimal for biomechanical stability [15].

These observations indicate that the 3D printing fixator has significant advantages in trunk bone surgery [16–18]. In this study, 66 clinical patients with rib fractures were divided into a non-3D printing group (control group) and a 3D printing group (intervention group) in a ratio of 1 : 1. The information including gender, age, incision length, number of surgical roots, bleeding volume, operation time, and intraoperative blood transfusion was paired with a series of SPSS analysis. The use of video-assisted thoracoscopic single-incision minimally invasive technology is expected to reduce the length of the incision in patients, shorten the operation time, reduce bleeding, postoperative intercostal neuralgia, and other complications, and ultimately reduce the mortality of trauma patients and improve the quality of life of patients.

## 2. Objective and Methods

Patients were prospectively and randomly selected and paired with similar parameters such as the number of fractured ribs, presence of other combined injuries, body mass index, and age and then divided into a three-dimensional printing group (intervention group) and a non-three-dimensional printing group (control group). From Tables 1 and 2, it can be seen that in terms of gender distribution in the control group, the majority of the samples were “men,” 24.0 in total, accounting for 72.73%. 69.70% of the samples in the intervention group were male. The proportion of female samples was 30.30%.  Figure 1 shows the mean of the intervention group. The mean ages of the two groups were 58.545 and 57.333.  Figure 2 shows the 3D printing fixator and wound indication.

## 3. Results and Discussion

As shown in Table 3, the paired *t*-test was used to interpret the data. It can be observed that among the three paired data sets, only one presented the difference (*p* < 0.05). The significance at the 0.01 level was found between the incision length/surgical root count in the control group and the incision length/surgical root count in the intervention group ((*t* = 4.232, *p* ≤ 0.001), and the difference embodied in the average incision length/surgical root count in the control group (4.86) was significantly higher than the average incision length/surgical root count in the intervention group (2.90). The intervention was effective. The data of the intervention group are further analyzed in Table 4.

As shown in Table 4, *n* = 25 because some data from patients were missed. Operation time, intraoperative blood transfusion, age, gender, and incision length/number of operation roots in the intervention group were chosen as independent variables, while the amount of bleeding was the dependent variable.

The value of the model pseudo-*R* formula was 0.107, indicating that the operation time, intraoperative blood transfusion, age, gender, and incision length/number of operation roots could explain the change of 10.7% in the bleeding volume. The formula is as follows: log (*u*) = 3.478 + 0.025∗ operation time + 0.000∗ intraoperative blood transfusion + 0.018∗ age + 0.089∗ gender + 0.027∗ incision length/number of operation roots. The final specific analysis shows the following.

The regression coefficient value of the operation time was 0.025, and the value was valid (*z* = 2.397, *p*=0.017) which meant that the operation time had a markable positive impact on the bleeding volume. And, an odds ratio (OR value) of 1.025 meant that the amount of bleeding changed (increased) by a factor of 1.025 when the surgical time added one unit.

The regression coefficient value of intraoperative blood transfusion was less than 0.001, and the value was valid (*z* = 11.066, *p* ≤ 0.001), which meant that intraoperative blood transfusion would have a markable positive impact on blood loss. And, an odds ratio (OR value) of 1.000 meant that the amount of bleeding changed (increased) by 1.000-fold when a unit was added to the intraoperative blood transfusion.

The regression coefficient for age was 0.018, and the value was valid (*z* = 7.921, *p* ≤ 0.001), It shows that age has a significant positive effect on bleeding volume. And, an odds ratio of 1.018 meant that the amount of bleeding changed (increased) by a factor of 1.018 with age.

The regression coefficient of gender was 0.089, but it was invalid (*z* = 1.919, *p*=0.055), indicating that gender had no effect on the amount of bleeding.

The regression coefficient value of incision length/number of surgical roots was 0.027, and it showed a prominent value at 0.05 level (*z* = 2.053, *p*=0.040 < 0.05), which meant that incision length/number of surgical roots had a huge positive impact on bleeding volume. And, an OR of 1.028 indicated a 1.028-fold change in bleeding volume with a one-unit increase in incision length/surgical root count.

According to the summary and analysis, four items including operation time, intraoperative blood transfusion, age, and incision length/operation root number all had significant positive impact on the bleeding volume. However, gender did not affect the amount of bleeding.

As shown in Table 5, only 25 complete cases could be analyzed. Incision length/number of surgical roots and operation time in the intervention group were observed as independent variables, while blood transfusion during the operation was the dependent variable. The formula was as follows: log (*Y*) = −2.806 − 0.400∗ incision length/number of surgical roots + 1.889∗ operation time. The regression coefficient value of incision length/number of surgical roots was −0.400, and there was a significant difference at the 0.05 level (*Z* = −2.436, *p*=0.015 < 0.05), which meant that incision length/number of surgical roots had a huge adverse impact on intraoperative blood transfusion. A ratio of 0.670 meant that the magnitude of the change (decrease) in intraoperative blood transfusion was 0.670-fold when the incision length/number of surgical roots was increased by one unit. The regression coefficient value of the operation time was 1.889, and the significance was shown at 0.01 level (*z* = 12.779, *p* ≤ 0.001), which meant that the operation time had a markable positive impact on the intraoperative blood transfusion. And, the odds ratio was 6.614, which meant the change (increase) in intraoperative blood transfusion was 6.614 times greater when the operation time added a unit. According to the above data, operation time had a markable positive impact on intraoperative blood transfusion and incision length/operation roots had a markable negative impact on intraoperative blood transfusion.

## 4. Conclusions

The results showed the following: the paired *t*-test was used to test the difference of experimental data. There was a significant difference of 0.01 between the incision length/root number in the intervention group and the incision length/surgical root number in the control group. The incision length/surgical root number in the intervention group was significantly lower than that in the control group. Surgical time, intraoperative blood transfusion, age, and incision length/root number in the intervention group had a significant positive impact on the amount of bleeding. Gender did not affect the amount of bleeding. A total of 1 item of operation time in the intervention group had a significant positive impact on intraoperative blood transfusion. The incision length/number of surgical roots in the intervention group had a great adverse impact on blood transfusion during the operation.

## Figures and Tables

**Figure 1:** Mean of the intervention group.

**Figure 2:** Surgical placement sequence of the 3D printing fixator and wound indication.

**Table 1:** Basic information results.

Project	Option	Number of people	Percentage	Cumulative percentage
Gender of the control group	Woman	9	27.27	27.27
	Man	24	72.73	100.00

Gender of the Intervention group	Woman	10	30.30	30.30
	Man	23	69.70	100.00

Total		33	100.0	100.0

**Table 2:** Basic indicators.

Name	Sample size	Minimum value	Maximum value	Average value	Median
Age of the control group	33	37.000	87.000	58.545	57.000
Age of the intervention group	33	32.000	73.000	57.333	56.000

**Table 3:** Analysis results of the paired *t*-test in the control group.

Name	Paired *t*-test (mean standard deviation)		Difference (pair 1 − pair 2)	*t*	*p*
	Pair 1	Pair 2			
Control group age paired with intervention group age	58.55 ± 10.58	57.33 ± 8.19	1.21	0.451	0.655
Control group incision length/number of surgical roots paired with intervention group incision length/number of surgical roots	4.86 ± 2.44	2.80 ± 1.16	2.07	4.232	≤0.001^*∗∗*^
Bleeding volume of the control group paired with bleeding volume of the intervention group	136.06 ± 141.99	131.21 ± 120.67	4.85	0.144	0.886

^∗∗^ *p* < 0.01.

**Table 4:** Poisson regression analysis of six factors (*n* = 25).

Project	Coefficient of regression	*Z* value	*p* value	OR value	OR value (95% CI)
Operation time	0.025	2.397	0.017	1.025	1.005∼1.047
Intraoperative blood transfusion	0.000	11.066	≤0.001	1.000	1.000∼1.000
Age	0.018	7.921	≤0.001	1.018	1.013∼1.022
Gender	0.089	1.919	0.055	1.093	0.998∼1.197
Incision length/number of operation roots	0.027	2.053	0.040	1.028	1.001∼1.055
Intercept	3.478	20.671	≤0.001	32.397	23.296∼45.053

Dependent variable: amount of bleeding; McFadden *R* formula: 0.107.

**Table 5:** Three-variable negative binomial regression analysis (*n* = 25).

Project	Coefficient of regression	*Z* value	*p* value	OR value	OR value (95% CI)
Intercept	−2.806	−3.419	≤0.001	0.060	0.012∼0.302
Incision length/number of operation roots	−0.400	−2.436	0.015	0.670	0.485∼0.925
Operation time	1.889	12.779	≤0.001	6.614	4.950∼8.836

Dependent variable: intraoperative blood transfusion; McFadden *R* formula: 0.173. ^∗∗^*p* < 0.01.

## Data Availability

All data supporting this work are included within the paper and the supplementary file.
